This article has been retracted.

# The Integration of Legal Education and Mental Health Education of College Students in the Contemporary Network Environment Facing the Cultivation of Civic Awareness

**DOI:** 10.1155/2022/4858156

**Published:** 2022-07-30

**Authors:** Yong Li, Chuang Bao, Ming Liu

**Affiliations:** University of International Business and Economics, Beijing 10029, China

## Abstract

Since the world entered the era of network information, the influence of the Internet has been expanding day by day, and today's college students are deeply affected by the network environment, which has also brought unprecedented challenges to the moral education work of colleges and universities. The rule of law education for college students is a key point for the comprehensive implementation of the strategy of governing the country by law. How to enhance the effectiveness and recognition of the rule of law education for college students has become an important task of higher education. Therefore, strengthening the legal education of college students is not only an inevitable choice to fully implement the rule of law but also a realistic requirement to improve the level of higher education and realize the all-round development of college students. College students' mental health education is an important part of the talent training system of colleges and universities, and in-depth exploration of the ideological and political laws of college students' mental health education courses is an inevitable requirement for implementing the fundamental task of Lide Shuren. College students' mental health education courses must be integrated into the ideological and political concepts of the curriculum, reflect the political orientation of ideological and political work, embody the law of educating people with morality as the first, and embody the practical purpose of psychology to pay attention to personality improvement. It is necessary to optimize the content of education and teaching, excavate the elements of ideological politics in the curriculum, enrich the resources of ideological politics in the curriculum, and explore a new way of reforming the ideological and political education curriculum for college students from the aspects of deeply planting family and national feelings, enhancing political identity, strengthening cultural self-confidence, cultivating Chinese temperament, clarifying the meaning of life, strengthening mission responsibility, enhancing civic awareness, and developing law-abiding habits. Strictly regulate the behavior of contemporary college students in the online environment, give full play to the role of legal education, and reduce the incidence of online incidents such as online fraud and cyber violence. This paper puts forward some problems in the current legal education of college students in China and points out the root causes of these problems. Methods for structural reform and advanced cultural construction based on social development are proposed. From a strategic point of view, it is believed that only by managing the reform of legal education and cultivating civic awareness can we completely solve various contradictions and problems among college students in the network environment and pave the way for the development of college students.

## 1. Introduction

Since the Fourth Plenary Session of the 18th Central Committee, under the background of vigorously promoting the construction of a country under the rule of law, my country has proposed more than 190 construction and reform tasks, and education is related to the future and development of the country. Construction is closely related. Colleges and universities, as important centers for cultivating talents, the rule of law education for college students is an extremely important part of the work of national rule of law education. The development of the rule of law education for college students is of great significance to the establishment of college students' legal thought, the improvement of legal awareness, the construction of a rule-of-law society, and the advancement of modernization [1]. Therefore, the ideological and political construction of college students' mental health education courses must follow the requirements of ideological and political work; highlight political orientation; unremittingly use Xi Jinping Thought on Socialism with Chinese Characteristics for a New Era to cast the soul and educate people; guide students to understand the world conditions, the national conditions, the party, and the people; enhance the “four consciousnesses”; strengthen the “four self-confidences”; and achieve “two safeguards.” If the mental health education curriculum abandons the political attribute, it will deviate from the requirements of the ideological and political construction of the curriculum of “guarding a good canal and planting a good responsibility field,” and it is difficult to form the effect of peering in the same direction and educating people in a coordinated manner.

The 18th National Congress of the Communist Party of China put forward the strategy of comprehensively promoting the rule of law. To comprehensively promote the rule of law, it is necessary to continuously improve the social and legal environment. To comprehensively promote the rule of law is to promote the spirit of the rule of law in the whole society, publicize the concept of the rule of law, develop the theory of the rule of law, apply the thinking of the rule of law, innovate the way of the rule of law, and make the spirit of the rule of law and the belief in the supremacy of the law become the common belief of Chinese citizens. This special group of college students is the backbone of future social construction and will have a profound impact on the process of legalization in our country. Because college students have the characteristics of plasticity and strong educability, it is determined that they will be the focus of civic education on the rule of law. Therefore, college students are bound to take the lead in becoming citizens under the rule of law [2, 3]. For a long time, the university legal education mainly adopts the “pay attention to classroom education, supplemented by practice” teaching mode; this mode is too eager although it can guide college students to quickly master the basic legal system and legal knowledge; however, the process of legal system attaches great importance to the teaching of knowledge theory, but ignores the teaching of concept, the construction of teachers, the depth of teaching, the practical activities, and classroom teaching, which leads to the unsatisfactory effect of legal education and makes it face greater difficulties.

Based on the above-discussed problems in legal education in colleges and universities, this paper investigates the status quo of legal education in college students through literature research and finds the main problems at present in the investigation process. In view of these problems, this paper puts forward corresponding solutions. Therefore, this paper is of great reference significance to grasp the historical responsibility and opportunity of the era of legal education in the new era and to construct and comprehensively promote the legal education and training system adapted to the rule of law.

## 2. Relevant Theoretical Basis

### 2.1. The Concept and Characteristics of Legal Education for College Students

Legal education is an important task in ideological and political education in the new period, but also with the development of the times, now this kind of security education has become a key point in the practice of ideological education and political work, and it is necessary to stabilize the situation and go deep into the popularization of the law, which is quite critical for college students, requiring students to carry out the development of a political and economic environment, to educate young descendants with the basic knowledge of socialist democracy and law, to let young people receive this kind of training and some education, and to strengthen the concept of the legal system. High school in the United States refers to all institutions engaged in higher education after the middle school stage, including all colleges and universities including vocational and technical colleges, junior colleges, and community colleges. Among them, junior colleges and community colleges have the nature of postsecondary education, which makes more Americans think that they are transitioning from secondary education to higher education, rather than pure colleges and universities. Therefore, the concept of “student” in American colleges and universities is relatively broad, and in a sense, it is more closely related to society. In my country, it is quite different. According to the “Higher Education Law of the People's Republic of China,” my country's higher education institutions generally refer to universities, independent colleges, and vocational colleges, including higher vocational schools and adult colleges. What is a “college student”? According to Article 37 of the “Measures for Handling Student Injury Accidents” by the Ministry of Education of the People's Republic of China, college students refer to those educated full-time in colleges and universities, including junior college students, undergraduate students, master students, and doctoral students. From the analysis of the scope of college students, college students in our country belong to a relatively closed educated group [4].

### 2.2. The Necessity of Legal Education for College Students

College students are the main group on the Internet, and the quality of the network environment will directly affect the mental health of college students and the formation of values and will also directly affect the reconstruction of the educational environment. Therefore, it is of great significance to strengthen the legal education of college students [5]. Network regulation should be done under the auspices of the government. Some students blindly pursue the realization of personal values, and the behavioral requirements of social life are generally not measured by whether the behavior is illegal. Thinking that the law is an after-the-fact remedy, as long as there is no accident, there is no need to learn legal knowledge, so the awareness of legal warning education is insufficient. Affected by the bad social atmosphere, students lack awareness of rules and disapprove of their own illegal behaviors. To deal with disputes and resolve conflicts, they will not hesitate to take risks and try the law by themselves [6–8].

### 2.3. The Social Value Theory Included in the Rule of Law Education for College Students

In a certain sense, the legal education of college students determines the degree and level of socialization of college students and determines whether the transition from students, builders, and successors can be smoothly realized; in today's society of advocating the legal system and pursuing civilization, the level of one's awareness of democracy and the legal system and the rigor of the concept of discipline determine the degree of realization of personal and social values. Education in the concept of the legal system is an important way to enhance college students' awareness of democracy and the legal system and their self-consciousness of discipline, and it is necessary to grasp it in a down-to-earth, well-grasped, and thorough manner, so as to help enhance the civilization of the whole society. Social value refers to the contributions and responsibilities that individuals make to meet the material and spiritual needs of society or others through their own and self-practice activities. Personal value refers to the discovery and creation of an individual or society in production and life to meet individual needs, which is the contribution of individual self-development and society to individual development. It includes the personal value of the individual and the personal value of the society and contributes to the freedom of different subjects to the individual. The social value and the personal value of the legal education of college students are related to each other, promote each other, and distinguish each other. Therefore, the relationship between the two is dialectically unified. Individuals constitute society, exist in society, and create society. The ontological basis of social history is people, and society is the totality of people who are interconnected based on common material production activities [8]. A society cannot be called a society without the reality of individuals and their activities, let alone development. Only through the education of the rule of law can we guide the thoughts and behaviors of individual college students, shape their legal personalities, stimulate their spirit of the rule of law, promote the improvement of college students' legal awareness and quality of the rule of law, and create dynamic undertakers and promoters for the implementation of the strategy of governing the country by law. The legal education of college students helps students develop legal awareness and the quality of the rule of law. This is also the personal value embodied by the legal education of college students. Only through the education of the rule of law in colleges and universities can the legal consciousness be internalized in the students' hearts, and the students' personal legal consciousness and quality of the rule of law can only be externalized through practical activities in society. Otherwise, the personal value of the legal education of college students is that only potential possible values exist. That is to say, only when the educated turn the legal awareness cultivated by the education of the rule of law into their own conscious actions to act on the society, promote the all-round development of the society, and thus realize the social value of the education of the rule of law, the personal value can be truly realized. Therefore, the social value and the personal value of legal education for college students are related to each other, promote each other, develop together, and are different from each other. The two are dialectically unified [9].

The social value and individual value of college students' legal education are interrelated, promoting, and developing together, which are different. In the network environment, the legal system education should be close to The Times characteristics, by building a legal system based on artificial intelligence network education platform, using data mining technology, ensure integration of the rule of law, case law education database, the use of experts and knowledge map to improve college students' legal quality, the overall system framework is shown in Figure 1.

### 2.4. Follow the Principle of Mental Health Education and Pay Attention to the Perfection of Personality

Psychology is the study of psychological phenomena, the exploration of psychological problems, and the revelation of the law of psychological development of science; the word psychology is derived from the Greek language, meaning the science of the soul; the core is to promote the integrity of human development and cultivate the perfection of students' inner personality. In 2011, the Ministry of Education issued the “Basic Requirements for the Teaching of Mental Health Education Courses for Students in Ordinary Colleges and Universities,” which clearly pointed out that the mental health education courses for college students “aim to enable students to clarify the standards and significance of mental health; enhance their awareness of self-mental health care and psychological crisis prevention; master and apply mental health knowledge; cultivate the self-cognitive ability, interpersonal communication ability, and self-regulation ability; effectively improve psychological quality; and promote the all-round development of students.” The objectives of the mental health education course for college students include education at the knowledge level, education at the skill level, and education at the level of self-awareness, so this course must use the theoretical knowledge and methods of psychology according to the physical and mental characteristics and growth laws of students to cultivate students' self-esteem and self-confidence, rational peace, positive health status, and correct behavior habits; realize the unity of knowledge and intention; promote the comprehensiveness, richness, and integrity of students' personalities; and adapt students to the changing social environment. If the mental health education curriculum ignores the cultivation of students' personalities, cannot resolve psychological problems such as students' psychological distress, emotional confusion, and emotional disorders in a timely manner, gives play to the guiding role of positive cognition, the stimulating role of positive emotions and emotions, and the forging role of positive will, enhances the temperature of humanistic care and focuses on the shaping of students' personality; it will deviate from the goal requirements of the course's ideological and political cultivation of sentiment, warm heart, and sound personality.

## 3. Online Legal Education and Mental Health Education Achievements for College Students

Contemporary college students, whether in the handling of individual consciousness and collective consciousness, in the balance of the online virtual world and real life, or in the choice of state responsibility and individual obligations, need to use civic consciousness to regulate and regulate informed intentions; otherwise, improper handling will greatly affect the mental health of college students. Therefore, in chapters such as “College Students' Interpersonal Communication, Love Pursuit, and Stress Management,” it is necessary to be good at integrating the educational content of civic awareness; take the cultivation of civic consciousness as an important starting point for promoting the mental health education of college students; use the situational teaching method to provide students with real-life scenarios; guide students to pay attention to strengthening civic awareness and legal awareness in the theoretical study of mental health; select typical cases; educate students in the practice of mental health; pay attention to transforming the requirements of the party and the state into the needs of college students' own growth; turn patriotic, dedicated, honest, and friendly civic consciousness into college students' daily code of conduct; promote the rationality and peace of college students' inner world; and develop good habits of abiding by the law. In order to understand the results of legal education and mental health education for contemporary college students in China, the research and analysis of college students was conducted.

### 3.1. Basic Situation

Through the above discussion of the concept and role of legal education in universities, the importance of promoting the legal education of college students can be basically understood. However, the achievements of online legal education can directly reflect the current situation of legal education in colleges and universities and the problems existing in the legal education of college students.

College students have a strong intention to conduct independent legal education through the Internet, which provides basic support for improving the content of college students' independent learning of the rule of law education. College students can learn the content of the rule of law education independently through the Internet, which is not limited by time and space. College students can learn the content of the rule of law education through the Internet anytime, anywhere, which greatly improves the autonomy of college students to participate in the activities of the rule of law education. In order to adjust the basic situation of college students' online legal education performance, the relevant data were obtained through research students understand the way to know the rule of law, as shown in Figure 2.

Most of the students believe that the Internet has a positive effect on the rule of law propaganda, and even 20% of the students believe that the Internet has a good effect on the rule of law education of college students, but 8% of the students believe that the Internet has no effect on promoting the rule of law education of college students; in addition, 442 52% of the students who participated in the survey chose “the effect is not obvious” for the question of “the role of the Internet in the education of the rule of law for college students”. The method is outdated and reduces the effect of using the Internet to promote the legal education of college students. At this stage, the effectiveness of using the Internet to carry out legal education in colleges and universities in my country needs to be strengthened. See Figures 3 and 4. In view of the above survey results, colleges and universities should re-examine the content of legal education on the basis of the goal of legal education, improve the publicity mode of legal education, and can combine the rule of law publicity with the main interests of college students while increasing the publicity but also can deepen the impression of the knowledge of the rule of law.

It is not very optimistic for college students to independently conduct legal education through the Internet. The Internet is an open space, and college students have more choices on the Internet [10]. College students are at a special age. They are physically mature but psychologically immature. Facing the temptation of the Internet, weak-willed college students will easily lack the awareness of self-education, resulting in wasted time on the Internet. In addition, through interviews with students, it is found that when practical legal issues are not involved, few students use the Internet to learn legal knowledge independently and conduct self-education on the rule of law in their spare time. The low enthusiasm of college students to study law is an important reason that restricts the effectiveness of online legal education for college students. The specific data are shown in Tables 1–3.

Conducted a survey on the specific situation of college students' use of the Internet and found that college students' use of the Internet mostly focused on life and entertainment, and less attention was paid to legal knowledge. The specific situation is shown in Figures 5 and 6

## 4. Ways to Improve the Rule of Law Education and Mental Health Education for College Students

With the vigorous development and rapid popularization of the network environment, China's college students have a poor concept of the legal system and a low legal quality, and it is difficult to meet the needs of a society ruled by law and the requirements of the reform of the market economic system. In order to improve the legal education of college students under the background of comprehensively raising civic awareness, we must first optimize the legal education environment in colleges and universities. The second is to accurately grasp the concept of legal education for college students, abandon the idea of utilitarian education, and continuously improve and perfect the educational model and approach. Focus on regulating the words and deeds of college students in the network environment.

### 4.1. Optimizing the Legal Education and Teaching Environment for College Students

The legal education environment for college students is an important part of the social legal environment. College students live and study in a specific campus environment, and the school's legal education environment has a great impact on the legal education of college students [11]. It is natural to impart legal theoretical knowledge to students through classroom teaching, but as an important part of the “two lessons,” the fundamental foothold of the “legal foundation” course lies in comprehensively cultivating and improving the legal quality of college students. On the one hand, it is necessary to implement “governing the school by law” and “educate people by law” and subtly affect the formation and improvement of students' legal awareness in the campus culture. On the other hand, in terms of school rules and disciplines, there should be “laws to follow” and “laws to follow”; especially for individual students' violations of laws and disciplines, they should be dealt with according to the rules, and a strong atmosphere of the rule of law should be created for students in daily life, to set an example for students to “have laws to abide by and act in accordance with the law” and provide a good campus legal education environment for cultivating college students' legal awareness [12].

### 4.2. Abandon the Idea of Utilitarian Education and Accurately Grasp the Concept of Legal Education for College Students

The rule of law education of college students is to cultivate students' legal awareness and spirit of the rule of law. We cannot emphasize the education of social value orientation and ignore the education of personal value orientation, so that students' legal education can become a law-abiding education for cultivating “obedience to the people,” and we can blindly emphasize personal value orientation education and ignore social value orientation education so that students' legal education can be cultivated. It is a “trickster” who only cares for his own self-interest, only considers himself without considering others, and tramples on the rights and public interests of others for the sake of personal interests. The order and harmonious development of society have become empty words. The rule of law education for college students should abandon the utilitarian educational thought and realize the dialectical unity of personal value orientation and social value orientation. The Fourth Plenary Session of the Eighteenth Party pointed out that it is necessary to promote the whole society to establish awareness of the rule of law and carry out in-depth publicity and education on the rule of law; the purpose is to cultivate citizens' legal awareness and the spirit of the rule of law. The spirit of the rule of law is a concept with very rich connotations. It is a synthesis of the values of the rule of law, such as fairness, equality, freedom, order, security, and the consistency of rights and obligations. It is the spiritual pillar of the construction of the rule of law system. It is a comprehensive proposition that integrates the spirit of human rights, the spirit of justice, the spirit of rationality, and the spirit of harmony. It is a scientific spirit formed by legal consciousness, legal thinking, legal psychology, and legal culture under the rule of law. It is also the guiding ideology and spiritual source of the practice of the rule of law. The cultivation of the legal spirit is not only the core goal of socialist rule of law construction but also the basis of legal education for college students [13].

### 4.3. Effective Ways and Modes of Legal Education for College Students

When college students receive legal education, the most important thing is the learning process. With the popularization of the network environment, the advantages of the network environment can be rationally used to more widely transfer the understanding points and values of legal education, which has a good effect on enhancing the legal concept of college students. The education of the rule of law for students in colleges and universities not only includes the education of basic legal theory and basic legal knowledge but also, more importantly, cultivates students' legal awareness and the spirit of the rule of law. According to actual needs and in combination with different majors in colleges and universities, some legal courses related to the majors studied by the students of the school can be opened, so as to cultivate students' conscious awareness and knowledge of law-abiding, law-abiding and usage. Compared with boring theoretical lectures, it is closer to life and more attractive. Therefore, it is necessary to break the single teaching mode of purely theoretical professors and carry out a variety of teaching activities; for example, organize students to watch legal dramas, set up legal elective courses, court access to campus, and legal sitcoms of campus life. Publicize legal knowledge through newspapers, lectures on legal knowledge and other channels; open the network legal lectures and create a good campus legal environment and legal atmosphere. Second, continue to strengthen the social practice of the rule of law. Practice is the only criterion for testing the truth, and practicality itself is the essential character of legal knowledge. Practical teaching occupies an extremely important position in the process of legal education and is an effective way to promote the formation of college students' legal awareness, legal spirit, and legal thinking. Practice is more persuasive than classroom teaching. The social practice teaching of legal education for college students should be based on the social legal environment, based on the actual social production and life, and through a large amount of information, and then multi-dimensionally and comprehensively display phenomena and problems and guide students through personal practice, independent analysis, and exploration of problems and phenomena. Behind, there lies the concept and value of rule of law [14].

The system of legal education cases needs to be strengthened. At this stage, the traditional legal education of college students who do not major in science in our country is the main way of “Ideological and Moral Cultivation and Legal Basis,” “Mao Zedong Thought and Introduction to the Theoretical System of Socialism with Chinese Characteristics,” “Situation and Policy,” and other courses. With the rapid development of society, the textbooks used in the courses are far from meeting the new teaching requirements. However, such public basic courses are offered uniformly by the state, and the content of the textbooks is also uniformly compiled by the Ministry of Education of the state. The updating and revision of textbooks often take a long time [15].

### 4.4. Strengthen the Construction of the Teachers' Team

The key to strengthening the construction of teachers is to strengthen the training of existing teachers. The training for educators mainly focuses on improving the legal literacy of educators and skills training in online course construction. First, teachers need to improve their own legal literacy. Due to their own limitations, educators reduce the effectiveness of online legal education for college students. Therefore, improving the legal literacy of educators plays an important role in enhancing the effectiveness of online legal education for college students [16]. To improve teachers' legal literacy lies in improving the ideological and political literacy, legal literacy, and lecturing ability to exist ideological and political educators. In view of the limitations of existing ideological and political educators in the legal profession, colleges and universities need to increase capital investment in legal education. The first is to regularly select and send ideological and political educators to participate in the training and advanced study of legal professional knowledge in a planned and targeted manner, so as to improve the legal literacy of legal educators from knowledge. At the same time, according to the teachers' own advantages and the existing conditions, teachers are encouraged to carry out further studies or to improve their academic qualifications in law. Second, colleges and universities can build judicial practice platforms to encourage educators to actively participate in judicial practice and academic exchanges. While expanding educators' horizons, they can also enhance educators' ability to use the law to solve problems and enrich educators' practical experience, so as to improve the educators of the rule of law theory and the purpose of the rule of law spirit. Secondly, to promote the online legal education of college students, the main body of education is college teachers. How teachers realize the integration of Internet and legal education is the key. Due to the limitations of teachers themselves and the lack of information technology, teachers use the Internet to promote the process of legal education for college students. Therefore, it is necessary to strengthen information technology training for teachers of legal education in colleges and universities, which is a requirement for college teachers in the context multiple times and an important way to promote online legal education for college students [17–19]. Information technology training for college teachers focuses on practicality, improving teachers' educational technology capabilities, allowing teachers to familiarize themselves with and understand the basic methods and means of integrating information technology and teaching, and master basic microlectures, MOOCs, and other networks. The principles and production methods of online classrooms will gradually introduce online courses into traditional legal education courses. Especially, legal professional teachers can use the technologies of online course construction such as microcourses and MOOCs, combined with the technical support provided by the school, to complete the recording of professional legal courses and gradually introduce online courses into traditional legal education courses. After the teachers of law majors truly realize the actual effect of the Internet on the education of the rule of law in universities and feel the practical benefits of the Internet to reduce their workload, they will be more active in the work of the Internet and the education of the rule of law for college students [20]. In addition, colleges and universities can also incorporate the effectiveness of rule of law education into teachers' year-end target assessment, formulate reward and punishment systems, and add or subtract points according to teachers' completion status, so as to increase teachers' attention to rule of law education and encourage educators to continue to work in rule of law education. Innovate teaching methods to improve the effectiveness of online legal education for college students.

### 4.5. Enhance Students' Political Identity and Home-Country Feelings

Mental health education originated in the West; its origin theory is rooted in the Western cultural value system; emphasizing scientificity, objectivity, and reproducibility, these important theoretical schools, ideological views, technical design, operational norms, and so on have played an important role in promoting the development of mental health education but inevitably infiltrated the Western discourse system, institutional characteristics, and cultural values. The seriousness and diversity of mental health problems of college students in the United States have become more and more prominent, and the US mental health service system is difficult to meet the rapidly growing demand for services because the federal government has less support for the mental health of college students, and the lack of higher education policies around topics such as reducing service costs, increasing service content, and improving service systems. According to the requirements of “suspension of classes without stopping teaching and suspension of classes without stopping learning,” the mental health education course for college students in China adopts the method of online teaching, strengthens the psychological counseling and humanistic care for college students in view of the difficult pain points of college students to cope with changes, and has received good results. Therefore, in “Overview of Mental Health,” attention should be paid to guide students to dialectically look at the development history of mental health education, the advantages, and characteristics of mental health education in our country to feel the superiority of the socialist system and enhance cultural identity.

## 5. Conclusion

College students' mental health education courses are directly related to the healthy growth of college students, involving the country's long-term peace and stability and national rejuvenation, and integrating the concept of curriculum thinking into the education and teaching of the curriculum is of great significance to innovating the mental health education model of college students and improving the pertinence and effectiveness of education and teaching and also puts forward higher requirements for professional teachers. The mental health education of college students must adhere to the student-centered and result-oriented education concept, constantly optimize the teaching content, deeply explore the ideological and political factors in the course teaching, strengthen the cooperative education consciousness, and enhance the cooperative education ability. Shape students' character, conduct, and taste, so that students with lofty aspirations, integrity, and ability, to become a mission worthy of the new generation. With the increasing influence of the Internet, college students account for half of the growing number of Internet users. They are deeply influenced by the network environment, whether from the perspective of thinking mode, language habit, or even from the perspective of learning and life style, which also brings unprecedented challenges to the moral education in colleges and universities. Cultivating and improving the legal quality of college students will greatly promote the process of building China's socialist legal system in the twenty-first century and is an inevitable requirement for governing the country according to law. This paper puts forward some problems in the current legal education of college students in China and points out the root causes of these problems. An approach to legal reform based on the network environment is proposed. To cultivate and improve the legal quality of college students, the teaching reform should be the leader, and the basic way to optimize the teaching links, make full use of modern media, strengthen the campus legal environment, strengthen the practical links, and expand the space for student development should be the basic way.

## Figures and Tables

**Figure 1:** Framework of network environment department legal education system based on artificial intelligence.

**Figure 2:** The way for college students to understand the law.

**Figure 3:** Pie chart of the role of the Internet in the education of the rule of law for college students.

**Figure 4:** Histogram of the effect of the Internet on the education of the rule of law for college students.

**Figure 5:** The main content ratio of college students using the Internet.

**Figure 6:** Distribution of the main content of college students using the Internet.

**Table 1:** Internet browsing content of the surveyed college students.

	Legal knowledge	Current news	Life entertainment	Others
People	36	114	144	56
Percentage	10.3	32.6	41.1	16.0

**Table 2:** Surveyed college students use the Internet to learn legal knowledge independently.

	Excellent	OK	No	No and lower
People	50	156	108	36
Percentage	14.3%	44.6%	30.9%	10.3%

**Table 3:** Surveyed college students watching online legal programs.

	Often	General	Occasional	Never
People	34	74	158	84
Percentage	9.7%	21.1%	45.1%	24.0%

## Data Availability

The labeled data set used to support the findings of this study is available from the corresponding author upon request.
